# Clinical Efficacy and Safety of Tumor Cytoreductive Surgery plus Hyperthermic Intraperitoneal Chemotherapy for Ovarian Cancer

This article has been retracted.

**DOI:** 10.1155/2023/6412679

**Published:** 2023-04-12

**Authors:** Huapeng Yu, Cuixia Xu, Qirong Li

**Affiliations:** ^1^Department of Obstetrics and Gynecology, Jinan Maternity and Child Care Hospital, No. 2 Jianguo Xiaojing 3rd Road, Shizhong, Jinan, Shandong, China; ^2^Laboratory, Qilu Hospital Huantai Branch, No. 2198, Huantai Avenue, Huantai Suo, Zibo, Shandong, China

## Abstract

**Objective:**

To assess the clinical efficacy and safety of cytoreductive surgery (CRS) plus hyperthermic intraperitoneal chemotherapy (HIPEC) for ovarian cancer.

**Methods:**

From April 2018 to November 2021, 66 patients with ovarian cancer were admitted to our hospital and randomly allocated to undergo intravenous chemotherapy following CRS (the observation group) or CRS with HIPEC (the experimental group) using a parallel randomized technique, with 33 cases in each group. Clinical effectiveness, intraoperative and postoperative recovery, VEGF level, T-lymphocyte subpopulation cell level, adverse events, and patient survival were all outcome metrics.

**Results:**

CRS plus HIPEC was associated with significantly higher clinical efficacy versus CRS alone (*P* < 0.05). The difference in the intraoperative bleeding and operative time between the two groups did not meet the statistical standard (*P* > 0.05). Patients in the experimental group experienced shorter postoperative chemotherapy and length of hospital stay than those in the observation group (*P* < 0.05). CRS plus HIPEC resulted in significantly lower levels of VEGFA, VEGFB, and VEGFC and higher levels of CD3+, CD4+, and CD3+/CD4+ than CRS alone (*P* < 0.05). The two groups of patients had a similar incidence of adverse events (*P* > 0.05). The experimental group showed a longer median survival (25 months) and a 1-year survival rate (79.55%) than the observation group (22 months, 49.56%) (log rank = 20.411, *P* < 0.05). A significantly lower 1-year recurrence rate was observed in the experimental group than in the observation group (*P* < 0.05).

**Conclusion:**

CRS plus HIPEC effectively improves the clinical efficacy of ovarian cancer patients, prolongs the survival of patients, and improves the level of VEGF and T-lymphocyte subpopulation cells, with a manageable safety. In addition, the treatment method can improve the therapeutic effect, reduce the toxic and side effects, and improve the immunity of the body, which is worthy of clinical promotion.

## 1. Introduction

Ovarian cancer is one of the three major malignant tumors in gynecology. The incidence of ovarian cancer in China ranks third after cervical cancer and uterine cancer. The incidence rate accounts for about 70% of malignant tumors, and it occurs in middle-aged and elderly women. The disease mostly occurs in the deep pelvic cavity, and the initial symptoms are relatively insidious. There is currently no effective screening method. Therefore, many patients have usually developed to the middle and advanced stages (stages III and IV) when they are identified. There are many types of ovarian tumors in women. In addition to the primary tumor, there will also be cases of metastases from other organs. It accounts for 10% of female malignant tumors and is the female tumor with the highest fatality rate [1]. At present, surgery and chemotherapy are the most commonly used methods for the treatment of ovarian cancer, but the recurrence rate after surgery is generally high. It has a greater impact and is often accompanied by bone marrow suppression and gastrointestinal symptoms. Studies have shown that if the recurrence time of platinum-resistant drugs is less than 6 months, the chemotherapy regimen generally does not choose platinum-containing single-agent regimens; platinum-sensitive recurrence time is greater than 6 months, and platinum-based combined chemotherapy regimens can be considered [2].

Currently, ovarian cancer patients are treated with tumor cytoreductive surgery (CRS), which allows for the precise removal of visible lesions [3]. According to clinical data, patients with advanced ovarian cancer typically have peritoneal lesions that cannot be entirely eliminated by CRS, resulting in postoperative recurrence and the need for subsequent adjuvant chemotherapy [4]. The low local drug concentration in the abdominal cavity of conventional systemic chemotherapy results in its poor eradication of residual tumor cells and therefore recurrence [5]. Hyperthermic intraperitoneal chemotherapy (HIPEC) is an emerging local chemotherapeutic technique in recent years, which is effective in targeting abdominal malignancies that are predisposed to metastasis [6]. HIPEC allows for the direct infusion of chemotherapeutic medications into the patient's peritoneal cavity, significantly increasing the concentration of local pharmaceuticals and therefore potentiating the pharmacological impact. This approach promotes chemotherapeutic medication penetration into tumor cells by increasing cell membrane permeability by local heating [7].

Many studies have shown that ovarian cancer patients after TCM adjuvant chemotherapy exhibited good outcomes. Traditional Chinese medicine believes that ovarian cancer belongs to the categories of “stony uterine mass” and “abdominal mass.” The cause is the deficiency of the righteous qi, which in turn causes the accumulation of damp heat and evil toxins, obstruction of the meridians and collaterals, and the formation of ovarian cancer. And after surgical treatment, a large amount of qi and blood in the body was wasted, the righteous qi became weaker, and the dampness and evil were infested. Therefore, the treatment should be to invigorate the righteous qi, promote the qi, and remove the blood stasis.

Herein, 66 patients with ovarian cancer admitted to our hospital from April 2018 to November 2021 were recruited to assess the clinical efficacy and safety of CRS plus HIPEC for ovarian cancer.

## 2. Materials and Methods

### 2.1. Participants

A total of 66 patients with ovarian cancer admitted to our hospital from April 2018 to November 2021 were recruited and assigned to receive intravenous chemotherapy after CRS (the observation group) or CRS plus HIPEC (the experimental group) via the parallel randomized method, with 33 cases in each group. This study was approved by the ethics committee of our hospital.

The randomization was carried out using an online web-based randomization tool (freely available at https://www.randomizer.org/). The randomization procedure and assignment were managed by an independent assistant who was not involved in screening or evaluation of the participants.

The original sample size calculation estimated that 30 patients in each group would be needed to detect a 3-point difference between groups in a 2-sided significance test with a power of 0.8 and an alpha error level of 0.05.

The study protocol and all amendments were approved by the appropriate ethics committee at each centre. The study was conducted in accordance with the protocol, its amendments, and standards of good clinical practice. All participants provided written informed consent before enrolment (KJ-KU20180605).

### 2.2. Inclusion and Exclusion Criteria

Inclusion criteria are as follows: (1) patients who were diagnosed with ovarian cancer by clinically relevant pathological tests; (2) patients who were tolerant to the treatment modality of this study; (3) patients whose residual lesions did not exceed 1 cm after CRS; (4) patients with a prognosis of survival >1 year and a KPS score >70; (5) patients without adhesions in the abdominal cavity; and (6) patients and family members were informed about the study and voluntarily participated in the study.

Exclusion criteria are as follows: (1) patients with other serious organ diseases; (2) patients with distant organ metastases; (3) patients with hematopoietic and immune dysfunction; (4) patients with psychiatric disorders or communication disorders; and (5) patients who dropped out, died, and those with poor compliance and difficulty in cooperating with this study.

### 2.3. Treatment Methods

Patients in both groups were treated with CRS. After routine general anesthesia, dissection was performed. The patient's abdomen was incised from the glabellar pubic bone to allow full exposure of the patient's operative field followed by resection of the ovarian in situ lesion, regional debridement of the patient's mural abdominal wall, and subsequent resection of the abdominal and intestinal organ lesions [8].

1. Patients in the observation group were treated with intravenous chemotherapy after CRS. Patients in the observation group received intravenous chemotherapy with paclitaxel injection (Chongqing Lemay Pharmaceutical Co., Ltd., State Drug Quotient H20054814) (175 mg/m^2^) combined with carboplatin for injection (Qilu Pharmaceutical Co., Ltd., State Drug Quotient H10920028, AUC = 5) from 7 to 14 d after satisfactory CRS. With every 3 weeks as 1 cycle of chemotherapy, a total of 6 cycles of treatment were performed [9].
2. Patients in the experimental group were treated with hyperthermic intraperitoneal chemotherapy (HIPEC) 7–13 d after CRS. Two perfusion tubes were placed in the left and right paracolic sulcus of the patient before the surgery, two drainage tubes were placed on the left and right pelvic floor of the patient, and the tubes flowing into the abdominal cavity were ≥25 cm. The treatment apparatus used was the BR-TRG-I body cavity thermal perfusion therapy system, and the perfusion fluid was 3000 mL of saline +50 mg/m^2^ of cisplatin (Qilu Pharmaceutical Co., Ltd., State Drug Quantifier H37021358). The perfusate was placed in the instrument and preheated to 43°C. The appropriate flow rate was adjusted with the perfusion maintained for 60–90 min. The perfusion fluid was infused through the perfusion tube and released through the drainage tube. The second intraperitoneal thermal perfusion was continued on the second postoperative day in the same manner and with the same dose, and the perfusion tube and drainage tube were removed the day after the end of perfusion [10]. The first course of intravenous chemotherapy was administered 14 d after surgery, and the chemotherapy regimen and duration of treatment were consistent with those of the observation group.

On the basis of the two groups, Yiqi Yangyin Decoction was given as an adjuvant therapy. Prescription: Jujube 10 g, *Platycodon grandiflorum* 10 g, *Polygonatum* 15 g, *Curcuma* 15 g, *Prunella vulgaris* 15 g, dried radix rehmanniae 20 g, Scrophulariaceae 20 g, *Sagittaria* 20 g, *Ligustrum lucidum* 20 g, *Astragalus* 35 g, and *Chinese yam* 25 g. The specific dose can be adjusted according to the symptoms. It was decocted in water, 1 dose/d, orally twice in the morning and evening, with 4 weeks as a course of treatment.

### 2.4. Outcome Measure

1. Clinical efficacy: clinical efficacy was classified into complete remission (CR), partial remission (PR), stable disease (SD), and progressive disease (PD) according to Response Evaluation Criteria in Solid Tumors (RECIST) 1.1.
2. Intraoperative and postoperative recovery: the intraoperative and postoperative recovery indices included intraoperative bleeding volume, operation time, chemotherapy time, and hospitalization time. All the above indexes were recorded by the relevant medical and nursing staff of our hospital.
3. Vascular endothelial growth factor (VEGF) levels: the levels of VEGFA, VEGFB, and VEGFC were determined before and 1 month after treatment by enzyme-linked immunosorbent assay.
4. T-lymphocyte subpopulation cell levels: the patients' peripheral blood CD3+, CD4+, and CD3+/CD4+ levels were determined before chemotherapy and 1 week after treatment using a FACS Calibur-type flow cytometer.
5. Adverse reactions and survival: The occurrence of adverse reactions during treatment and 1-year survival was recorded for both groups of patients. Adverse reaction conditions included wound infection, venous thrombosis, and bone marrow suppression.

### 2.5. Statistical Analysis

SPSS22.0 was used for data management and analyses. The measurement data were expressed as mean ± standard deviation ($\bar{x}\pm s$) and analyzed using the *t*-test. The count data were expressed as rates (%) and subject to the chi-square test. The Kaplan–Meier method was used to calculate the median survival time and the survival rate and plot the survival curve, and the Log-rank test was used to analyze the survival of the two groups. *P* < 0.05 was used as a cut-off for statistical significance.

## 3. Results

### 3.1. Patient Characteristics

This study comprised 66 ovarian cancer patients who were randomly assigned to two groups: observation (*n* = 33) or experimental (*n* = 33) using the parallel randomized controlled trial technique. Patients in the observation group were aged 27–74 (58.62 ± 5.73) years, with a BMI of 14.2–33.8 (23.27 ± 4.29) kg/m^2^. There were 18 primary and 15 recurrent tumor types, 21 plasmacytic, 4 mucinous, 5 mixed and 3 other pathological types, 16 lymph node metastases, and 17 non-lymph node metastases. Patients in the experimental group were aged 26–76 (58.74 ± 5.69) years, with a BMI of 14.1–33.6 (23.31 ± 4.34) kg/m^2^. There were 189 primary and 14 recurrent tumor types, 19 plasmacytic, 7 mucinous, 7 mixed and 5 other pathological types, 15 lymph node metastases, and 18 non-lymph node metastases. The patient characteristics between the two groups were comparable (*P* > 0.05). (Table 1).

### 3.2. Clinical Efficacy

In the observation group, there were 7 cases of CR, 5 cases of PR, 10 cases of SD, and 11 cases of PD, and the overall response rate (ORR) was 66.67% (22/33). In the experimental group, there were 9 cases of CR, 14 cases of PR, 7 cases of SD, and 3 cases of PD, with an ORR of 90.90% (30/33). CRS plus HIPEC was associated with significantly higher clinical efficacy versus CRS alone (*P* < 0.05). (Figure 1).

### 3.3. Intraoperative and Postoperative Recovery

The difference in intraoperative hemorrhage and operational time between the two groups was not statistically significant. Patients in the experimental group had shorter postoperative chemotherapy and hospital stays than those in the control group (*P* < 0.05) (Table 2).

### 3.4. VEGF Levels

Before treatment, there was no significant difference in the levels of VEGFA, VEGFB, and VEGFC between the two groups. CRS combined with HIPEC resulted in much lower VEGFA, VEGFB, and VEGFC levels than CRS alone (*P* < 0.05) (Table 3).

### 3.5. T-Lymphocyte Subpopulation Cell Levels

Before treatment, there were no significant differences in CD3+, CD4+, or CD3+/CD4+ levels between the two groups (*P* > 0.05). CRS plus HIPEC was associated with significantly higher levels of CD3+, CD4+, and CD3+/CD4+ than CRS alone (*P* < 0.05) (Table 4).

### 3.6. Adverse Events and Survival

The incidence of adverse reactions was 27.3% (9/33) in the observation group and 21.2% (7/33) in the experimental group. The two groups of patients had a similar incidence of adverse events (*P* < 0.05). The experimental group showed a longer median survival (25 months) and 1-year survival rate (79.55%) than the observation group (22 months, 49.56%) (log rank = 20.411 and *P* < 0.05). A significantly lower 1-year recurrence rate was observed in the experimental group than in the observation group (*P* < 0.05) (Figures 2 and 3).

## 4. Discussion

With the rapid development of economy in recent years, the pace of people's life has accelerated, the pressure on women in all aspects of life and work has increased, environmental pollution has aggravated, the number of new cases of ovarian cancer is increasing year by year, and it has become one of the more common malignant tumors in the female reproductive system, with a fatality rate of over 60% [11, 12]. Ovarian cancer is relatively insidious and difficult to detect and diagnose and provide clinical intervention in the early stage. Most patients are already in the middle and late stages when they go to the doctor. Cancer cells usually spread to various parts such as the uterus and appendages, making treatment more difficult and ineffective. The anatomical position of the ovary is special, and the pelvic and abdominal cavities are at risk of diffuse implant metastasis during surgery [13, 14]. Most patients have advanced ovarian cancer by the time of diagnosis, and advanced ovarian cancer is characterized by abdominal implantation and metastasis; therefore, adjuvant therapy plus chemotherapy is required after CRS [15]. Conventional intravenous chemotherapy is ineffective in killing and removing residual lesions and free tumor cells, which is associated with an increased risk of ovarian cancer recurrence [16]. HIPEC is a new type of chemotherapy based on the different tolerance of tumor cells and normal cells to temperature, and HIPEC causes irreversible damage to tumor cells at 43°C [17]. The HIPEC technique improves the activity of chemotherapeutic drugs, promotes the intertissue penetration of drugs, and interferes with the metabolism of tumor cells, which well inhibits ovarian cancer cells from developing distant metastases [18]. High-volume peritoneal perfusion causes secondary elimination of free tumor cells in the pelvic and abdominal cavities and effectively reduces the risk of subsequent recurrence [19].

In the present study, the experimental group had a higher ORR and shorter duration of postoperative chemotherapy, length of hospital stay, and a lower 1-year postoperative disease recurrence rate than the observation group, suggesting that HIPEC after CRS effectively enhances the clinical outcome and postoperative recovery of ovarian cancer patients and reduces their risk of disease recurrence. This is because intraperitoneal hyperthermic perfusion chemotherapy can greatly increase the tissue penetration of chemotherapeutic drugs and improve its anti-tumor effect; it can also kill heat-sensitive G0 cells, resulting in clinical benefits [20]. VEGF is a provascular endothelial cell growth factor including several isoforms; VEGFA and VEGFB have the effect of inducing neovascularization, while VEGFC induces lymphangiogenesis. Studies have confirmed that neovascularization provides support for the survival and proliferation of tumor cells, while the generation of lymphatic vessels provides conditions for the metastasis of tumor cells. Ghirardi et al. [21] showed that the thermal effect of HIPEC paired with chemotherapeutic drugs effectively inhibited the neovascularization of tumor tissues and also enhanced the sensitivity of tumor cells to chemotherapeutic drugs. In the present study, the levels of VEGFA, VEGFB, and VEGFC in the experimental group of patients after treatment were lower than those in the observation group of patients, indicating that CRS plus HIPEC could further inhibit tumor neovascularization and tumor local lymphangiogenesis in ovarian cancer patients, which is consistent with the findings of Ghirardi et al. This is because the thermal effect and chemotherapeutic drugs can synergistically inhibit tumor tissue neovascularization and at the same time increase the sensitivity of tumor cells to chemotherapeutic drugs, resulting in degeneration and necrosis of tumor tissue due to hypoxia, acidosis, and nutritional disorders [22].

Clinical studies have revealed a strong correlation between the level of T-cell differentiation and immune function, resulting in low immune function. Th1 cells have a regulatory immune role, and their elevated levels decrease the recognition of tumors by immune cells. Th2 cells have cytotoxic effects and can recognize and kill tumor cells [23]. In the present study, the CD3+, CD4+, and CD3+/CD4+ levels of patients in the experimental group were higher than those in the observation group after treatment, indicating that CRS plus HIPEC could better enhance the immune function of ovarian cancer patients. The clinical mechanism of action of CRS plus HIPEC to enhance immune function has not yet been clarified [24]. This is because the thermal effect can enhance the body's immune function, stimulate specific immune responses, and then enhance its own anti-tumor effect.

HIPEC increases the concentration of intraperitoneal drugs exponentially to promote apoptosis of cancer cells on the basis of the high-temperature killing of tumor cells [25], while some drugs in HIPEC do not enter the body circulation directly, thereby reducing the toxic side effects of chemotherapy drugs on patients' kidneys and gastrointestinal tract [26]. In the present study, there was no significant difference in the incidence of adverse reactions and survival between the two groups of patients. The median survival time was significantly longer in the experimental group (25 months) than in the observation group (22 months), and the 1-year survival rate was significantly higher in the experimental group (79.55%) than in the observation group (49.56%). This is similar to the results of the study by Xie et al. [27, 28] who used cisplatin for HIPEC, in which the prognosis and the survival rate of patients treated with HIPEC were better than those without HIPEC, indicating that the HIPEC features manageable safety in the treatment of ovarian cancer.

In addition, we also used traditional Chinese medicine treatment after surgery. Traditional Chinese medicine adjuvant chemotherapy has relatively good clinical feedback in the treatment of ovarian cancer, which can improve the treatment effect and reduce the toxic and side effects caused by chemotherapy and the impact on T-cell subsets. Chinese medicine believes that after chemotherapy, a large amount of qi, blood, and body fluids will be consumed, and the human body will be in a state of weakened yin and yang, which is easy to form the symptoms of deficiency and excess of phlegm coagulation, qi stagnation, stasis, and toxin. The main functions of Yiqi Yangyin Decoction are to clear away heat, detoxify, disperse knots, and nourish yin. *Astragalus* in the recipe can invigorate Qi, strengthen the spleen, and reduce swelling and diuresis; Chinese yam can invigorate the spleen and kidney, improve eyesight, and soothe the nerves; *Ligustrum lucidum* can nourish the liver and the kidney; *Curcuma lucidum* can promote Qi, relieve pain, eliminate accumulation, and disperse knots; Scrophulariaceae can nourish yin and cool blood, clear heat, and detoxify; *Sagittaria* and *Prunella vulgaris* can clear heat, detoxify, and disperse knots to eliminate carbuncle. The combination of the two drugs can accelerate the apoptosis of tumor cells. The combination of various medicines has the effects of clearing away heat, detoxifying, nourishing qi and yin, dispersing knots, and strengthening the body, thereby promoting the body to secrete immune factors, and has a good effect on adjuvant chemotherapy.

However, this study has the following limitations: (1) the observation time of this subject is short, and the number of cases collected is small; (2) due to the limitation of scientific research time and scientific research funds, this subject failed to study the mechanism of action of the drug through animal experiments; and (3) the follow-up time of this experiment is short, and there is no evaluation of the long-term effects of patients after surgery. Future studies with a larger sample size and long-term follow-up will be conducted to obtain more reliable data.

## 5. Conclusion

CRS plus HIPEC effectively improves the clinical efficacy of ovarian cancer patients, prolongs the survival of patients, and improves the level of VEGF and T-lymphocyte subpopulation cells, with a manageable safety. In addition, Yiqi Yangyin Decoction has a good therapeutic effect on patients with ovarian cancer after chemotherapy, which can reduce toxic and side effects and improve immune function, which is worthy of clinical promotion.

## Figures and Tables

**Figure 1:** Clinical efficacy (*n* (%)). *Note.*^*∗*^indicates *P* < 0.05.

**Figure 2:** Adverse events (n(%)). *Note.*^*∗*^indicates *P* < 0.05. ^*#*^indicates *P* > 0.05.

**Figure 3:** The Kaplan–Meier survival curve.

**Table 1:** Patients' characteristics ($\bar{x}\pm s$, *n* (%)).

	Observation (*n* = 33)	Experimental (*n* = 33)	*t*/*x*^2^	*P* value
Age (years)	27–74	26–76		
Mean age (years)	58.62 ± 5.73	58.74 ± 5.69	−0.085	0.933
BMI (kg/m^2^)	14.2–33.8	14.1–33.6		
Mean BMI (kg/m^2^)	23.27 ± 4.29	23.31 ± 4.34	−0.038	0.97
Tumor type			0.062	0.804
Primary	18	19		
Recurrent	15	14		
Pathological type				
Plasma type	21	19	0.254	0.614
Mucus type	4	7	0.982	0.322
Mixed type	5	7	0.407	0.523
Others	3	5	0.569	0.451
Lymph node metastasis			0.061	0.805
Yes	16	15		
No	17	18		

**Table 2:** Intraoperative and postoperative recovery ($\bar{x}\pm s$).

Indices	Observation (*n* = 33)	Experimental (*n* = 33)	*t*-value	*P* value
Intraoperative bleeding volume (mL)	379.68 ± 38.47	378.26 ± 39.14	0.149	0.882
Operative time (min)	101.36 ± 11.27	99.67 ± 10.35	0.634	0.528
Chemotherapy time (d)	8.97 ± 0.93	7.02 ± 0.72	9.524	<0.001
Hospitalization time (d)	11.39 ± 1.29	9.11 ± 0.87	8.418	<0.001

**Table 3:** VEGF levels ($\bar{x}\pm s$, *µ*g/L).

Timepoint	Indices	Observation (*n* = 33)	Experimental (*n* = 33)	*t*-value	*P* value
Before treatment	VEGFA	291.34 ± 40.11	289.68 ± 39.73	0.169	0.866
	VEGFB	365.87 ± 44.18	367.11 ± 40.68	−0.119	0.906
	VEGFC	232.42 ± 38.92	229.78 ± 41.74	0.266	0.791

After treatment	VEGFA	186.71 ± 21.39^*∗*^	102.37 ± 16.88^*∗*^	17.781	<0.001
	VEGFB	291.28 ± 23.14^*∗*^	143.84 ± 20.73^*∗*^	27.262	<0.001
	VEGFC	189.94 ± 25.21^*∗*^	92.46 ± 20.69^*∗*^	17.17	<0.001

*Note.* ^*∗*^indicates *P* < 0.05 when compared with pretreatment.

**Table 4:** T-lymphocyte subpopulation cell levels ($\bar{x}\pm s$).

Timepoint	Indices	Observation (*n* = 33)	Experimental (*n* = 33)	*t-value*	*P value*
Before treatment	CD3+ (%)	30.47 ± 3.19	30.33 ± 3.15	0.179	0.858
	CD4+ (%)	26.78 ± 2.74	26.75 ± 2.72	0.045	0.946
	CD3+/CD4+	1.13 ± 0.17	1.15 ± 0.14	−0.522	0.603

After treatment	CD3+ (%)	33.17 ± 3.44^*∗*^	35.59 ± 3.65^*∗*^	−2.772	0.007
	CD4+ (%)	34.08 ± 3.58^*∗*^	36.19 ± 3.73^*∗*^	−2.344	0.022
	CD3+/CD4+	0.85 ± 0.08^*∗*^	0.94 ± 0.11^*∗*^	−3.801	<0.001

*Note.* ^*∗*^indicates *P* < 0.05 when compared with pretreatment.

## Data Availability

All data generated or analyzed during this study are included within this published article.
